# MicroRNA-203 suppresses gastric cancer growth by targeting PIBF1/Akt signaling

This article has been retracted.

**DOI:** 10.1186/s13046-016-0323-1

**Published:** 2016-03-15

**Authors:** Shao-Jun Chu, Ge Wang, Peng-Fei Zhang, Rui Zhang, Yan-Xia Huang, Yun-Min Lu, Wei Da, Qun Sun, Jing Zhang, Jin-Shui Zhu

**Affiliations:** Department of Gerontology, Shanghai Jiao Tong University Affiliated Shanghai Sixth People’s Hospital, Shanghai, 200233 China; Department of Gastroenterology, Shanghai Jiao Tong University Affiliated Shanghai Sixth People’s Hospital, Yishan Road No. 600, Shanghai, 200233 China

**Keywords:** miRNA-203, Growth, Gastric cancer, PIBF1, Akt

## Abstract

**Background:**

MicroRNAs (miRNAs) have been proved involved in many tumorigenic behaviors including tumor growth. But, the clinical significance and functions of miRNA-203 in gastric cancer (GC) remain elusive.

**Results:**

Decreased expression of miRNA-203 was correlated with tumor size, poor prognosis and recurrence in GC patients. Overexpression of miR-203 or knockdown of its target progesterone immunomodulatory binding factor 1 (PIBF1) inhibited GC growth in vitro and in vivo, while miR-203 knockdown promoted GC proliferation. In addition, PIBF1 overexpression attenuated the inhibitory effects of miR-203 on GC growth and enhanced that effect on p-Akt expression.

**Conclusions:**

MiR-203 as a tumor biomarker suppresses GC growth through targeting the PIBF1/Akt signaling, suggesting that it may have the important therapeutic potential for the treatment of GC.

**Electronic supplementary material:**

The online version of this article (doi:10.1186/s13046-016-0323-1) contains supplementary material, which is available to authorized users.

## Background

Gastric carcinoma (GC) is the third leading causes of cancer-related deaths in the worldwide [1]. It is known that high recurrence rate and rapid tumor growth have become the major disturbance to improve the survival of GC. Though, the treatment strategies of GC, such as surgical resection and chemotherapy, are effective way to increase therapeutic outcome, GC patients still have high risk and mortality [2]. Mounting evidence shows that many oncogenes or anti-oncogenes are associated with GC development and progression. However, the underlying molecular mechanisms of GC are still poorly understood. Thus, identification of the biomarkers related to GC growth is urgently needed.

MicroRNAs as small noncoding RNAs of approximately 18-25 nucleotides are involved in regulation of cancer development and progression in various types of cancers, acting as either oncogenes or tumor suppressor genes [3]. Previous studies have reported that miR-144, miR-1266, miR-206, MiR-133b, and miR-26a function as tumor suppressors in GC, while miR-196a/196b and miR-301a function as the oncogenes in GC and colorectal cancer [4–10]. Circulating miR-203 represents the potential biomarker for evaluating the lymphatic node status of cervical cancer patients [11] and regulates epithelial to mesenchymal transition [12]. MiR-203 inhibits the proliferation and migration in esophageal cancer cells [13] and decreases nasopharyngeal carcinoma radio resistance by targeting IL-8/Akt signaling [14]. But, few studies indicate that upregulation of miR-203 enhances the malignancy of hypopharyngeal squamous cell carcinoma [15]. The correlation of miR-203 expression with GC has not been reported.

To confirm the relationship of miR-203 expression with GC growth, we previously identified differentially expressed miRNAs between GC tissues and adjacent non-tumor tissues (ANTT). MiRNA expression profiles showed that miR-203 was significantly downregulated in GC tissues. It has been manifested that miR-203 is abnormally expressed in different tumors including breast cancer, GC, cervical cancer, melanoma, human glioma, esophageal cancer and lung cancer, and its down-regulation is implicated in promoting cell proliferation, invasion and metastasis in multiple cancer cells [16–25]. But, the contribution of miR-203 to GC growth is still unclear.

In the present study, our studies demonstrated that decreased expression of miR-203 predicted poor prognosis and recurrence in GC patients and miR-203 overexpression or knockdown of its target PIBF1 inhibited cell proliferation and the colony formation of GC cells by inhibition of Akt signaling. Our findings suggested that miR-203 might function as the tumor suppressor in human GC growth by targeting the PIBF1/Akt signaling.

## Methods

### Materials

Human GC tissues and the ANTT were collected from Shanghai Jiao Tong University affiliated Shanghai Sixth People’s Hospital. GES-1 and GC cell lines (HGC-27, MKN-28, MKN-45, MGC-803, AGS, SGC-7901 and BGC-823) used in these experiments were from Laboratory of Gastroenterology of Shanghai Sixth People’s Hospital. Lentivirus-mediated miR-203 overexpression, miR-203 shRNA or PIBF1 shRNA vector, negative control vector (NC), and virion-packaging elements were purchased from Genechem (Shanghai, PR, China); All antibodies used in this study were purchased from Cell Signaling Technologies (Beverly, MA, USA).

### Drugs and reagents

Dulbecco’s Modified Eagle medium (DMEM) and fetal bovine serum (FBS) were from Thermo Fisher Scientific Inc (Waltham, MA, USA); 3-(4,5)-dimethylthiahiazo (-z-yl)-3,5- di-phenytetrazoliumromide (MTT) was from Dingguo biology (Shanghai, China); TRIzol Reagent and Lipofectamine 2000 were from Invitrogen (Carlsbad, CA, USA); M-MLV Reverse Transcriptase was from Promega (Madison, WI, USA); SYBR Green Master Mixture was from Takara (Otsu, Japan); RNase A was from KeyGEN biology (Nanjing, China). ECL-PLUS/Kit was from GE Healthcare (Piscataway, NJ, USA).

### Clinical samples and data

Tumor tissues were collected from biopsy samples undergoing resection of the primary GC in a total of 100 consecutive cases admitted in our hospital from January 2007 to September 2015. The baseline characteristics of the patients before neo-adjuvant chemotherapy were summarized. Follow-up studies included physical examination, laboratory analysis, and computed tomography if necessary. Overall survival (OS) was defined as the interval between the dates of surgery and death. The study was approved by Medical Ethics Committee of Shanghai Jiao Tong University and written informed consent was obtained from the patients or their parents before sample collection.

### MiRNA microarray analysis

MiRNAs were extracted from 3 pairs of GC tissues and corresponding ANTT samples and hybridized on miRNA microarray chip containing human miRNA probes found in the miRNA Registry (http://www.mirbase.org/ accessed miRBase R16.0, Sept 2010). Microarray chip analysis was performed by KANGCHEM (Shanghai, PR, China).

### Immunohistochemical staining

Anti-PIBF1 antibody was used for immunohistochemical (IHC) detection of the expression of PIBF1 protein in GC tissues, whose sections were processed for IHC analysis. For anti-PIBF1 IHC, unmasking was performed with 10 mM sodium citrate buffer, pH 6.0, at 90 °C for 30 min. Sections were incubated in 0.03 % hydrogen peroxide for 10 min at room temperature, to remove endogenous peroxidase activity, and then in blocking serum for 30 min at room temperature. Anti-PIBF1 antibody was used at a dilution of 1:200. The antibody was incubated overnight at 4 °C. Sections were then washed three times for 5 min in PBS. Non-specific staining was blocked with 0.5 % casein and 5 % normal serum for 30 min at room temperature. Finally, staining was developed using diaminobenzidine substrate, and sections were counterstained with hematoxylin. Normal serum or PBS was used to replace PIBF1 antibody in negative control. PIBF1 expression was semi-quantitatively counted as the total IHC staining scores [26].

### Construction of vectors

A fragment of miR-203 was generated by using the following primers: sense, 5’- GAATTCGGCGTGTCCCTTGACCC-3’ and antisense, 5’- CTCGAGGGAGGAGGGGAATGTGCA-3’ and inserted into the pMD-18 T vector with a green fluorescent protein reporter gene within the *E*coRI/*X*hoI restriction sites. The aforementioned miR-203 plasmid pCDNA3-GFP was transfected into 293 T cells, and the lentiviral particle-enriched supernatant was obtained 48 h later. A scrambled sequence (5’-TTCTCCGAACGTGTCACGT-3’), which had no homology with the human gene, was used as a scrambled negative control.

### Cell culture and lentiviral infections

GC cells were cultured in DMEM medium supplemented with 10 % heat-inactivated FBS, 100 U/ml of penicillin, and 100 μg/ml of streptomycin. Cells in this medium were placed in a humidified atmosphere containing 5 % CO_2_ at 37 °C. On the day of transduction, GC cells were replated at 5 × 10^4^ cells/well in 24-well plates containing serum-free growth medium with polybrene (5 mg/ml). Cells were transfected with recombinant experimental virus or control virus, and cultured at 37 °C and 5 % CO2 for 4 h. Then supernatant was discarded and serum containing growth medium was added. Positive and stable transfectants were selected and expanded for further study.

### Quantitative real-time PCR

To quantitatively confirm the mRNA expression levels of miR-203 in GC tissues, real-time PCR was performed. Total RNA was extracted from each clone using TRIzol according to the manufacturer’s protocol. Reverse transcription was carried out using M-MLV and cDNA amplification was performed using the SYBR Green Master Mix kit according to the manufacturer’s guidelines. Human glyceraldehyde-3-phosphate dehydrogenase (GAPDH) gene or U6 was used as an endogenous control. Data were analyzed using the comparative Ct method (2^-△△Ct^). Three separate experiments were performed for each clone.

### Western blot analysis

GC cells were harvested and extracted using lysis buffer (Tris-HCl, SDS, Mercaptoethanol, Glycerol). Cell extracts were boiled for 5 min in loading buffer and then equal amount of cell extracts were separated on 15 % SDS-PAGE gels. Separated protein bands were transferred into polyvinylidene fluoride (PVDF) membranes and the membranes were blocked in 5 % skim milk powder. The primary antibodies were diluted according to the instructions of antibodies and incubated overnight at 4 °C. Then, horseradish peroxidase-linked secondary antibodies were added at a dilution ratio of 1:1000, and incubated at room temperature for 2 h. The membranes were washed with PBS for three times and the immunoreactive bands were visualized using ECL-PLUS/Kit according to the kit’s instruction. The relative protein level in different groups was normalized to Tubulin concentration. Three separate experiments were performed for each clone.

### Cell viability assay

Cell proliferation was analyzed using the MTT assay. Briefly, GC cells transfected with miR-203 or PIBF1 shRNA were incubated in 96-well-plates at a density of 1 × 10^5^ cells per well with DMEM medium supplemented with 10 % FBS. Cells were treated with 20 μl of MTT dye and subsequently incubated with 150 μl of DMSO for 5 min. The color reaction was measured at 570 nm using an Enzyme Immunoassay Analyzer (Bio-Rad, Hercules, CA). The proliferation activity was calculated for each clone.

### Colony formation assay

2 × DMEM containing 20 % FBS and 5 × 10^3^ cells was mixed with equal volume of 0.7 % agarose and immediately plated in 6-well plates containing an underlayer of 0.5 % agarose made in 1× DMEM supplemented with 10 % FBS. The plates were cultured at 37 °C under 5 % CO2 for 5 to 7 days. Surviving colonies were counted and photographed with a Qimaging Micropublisher 5.0 RTV microscope camera (Olympus, Tokyo, Japan).

### Dual-luciferase reporter assay

HGC-27 and MGC-823 cells were seeded into 24- well plates. After 18 ~ 24 h incubation, 1 mg pmirGLO report vector carrying wild type 3’-UTR or mutated 3’-UTR of miR-203 targets was co-transfected with 100 pmol negative control or miR-203 into the GC cells using X-tremeGENE reagent. 48 h after transfection, fiefl and Renilla luciferase activities were measured with a Dual-Luciferase Reporter System (Promega). PmirGLO report vector was used as a positive control.

### Animal experiments

Six-week-old female immune-deficient nude mice (BALB/c-nu) were bred at the laboratory animal facility (Institute of Chinese Academy of Sciences, Shanghai, China), and were housed individually in microisolator ventilated cages with free access to water and food. All experimental procedures were performed according to the regulations and internal biosafety and bioethics guidelines of Shanghai Jiao Tong University and the Shanghai Municipal Science and Technology Commission. Mice were injected subcutaneously with 1 × 10^5^ GC HGC-27 cells in 50 μl of PBS pre-mixed with an equal volume of Matrigel matrix (Becton-Dickinson). Mice were monitored daily and developed a subcutaneous tumor. When the tumor size reached 5 mm in length, they were surgically removed, cut into 1-2 mm3 pieces, and re-seeded individually into other mice. When tumor size reached 5 mm in length, the mice were randomly classified as miR-NC group and miR-203 group. 15 μl of lentivirus was injected into subcutaneous tumors using a multi-site injection format. Injections were repeated every other day after initial treatment. The tumor volume every three days was measured with a caliper, using the formula: volume = (length × width)2/2.

### Statistical analysis

SPSS 20.0 was used for the statistical analysis. All of the values were recorded as the mean ± SEM from at least 3 independent experiments. Kruskal-Wallis H test and Chi-square test were used to analyse the expression rate in all groups. One-way analysis of variance (ANOVA) was used to analyze the differences between groups. The LSD method of multiple comparisons was used when the probability for ANOVA was statistically significant. Statistical significance was set at *P* < 0.05.

## Result

### MiR-203 is downregulated in human GC tissue

The miRNA expression profiles showed that miR-203 was down-regulated in GC tissues, compared to the ANTT (Fig. 1a). To validate this result, we accomplished the quantitative Real-time PCR in 100 cases of GC tissues and ANTT. Compared with the 41 cases of ANTT, miR-203 was markedly lowly-expressed (more than 2-fold; i.e., log2 [fold change] >1) in 59 cases of GC (*P* < 0.01; Fig. 1b). These data suggested that aberrant expression of miR-203 was a frequent event in human GC tissues. Consistent with the miRNA array data, the expression level of miR-203 was negatively correlated with the tumor size in GC patients (Fig. 1c).

**Fig. 1:** MiR-203 was downregulated in human GC tissue and was correlated with tumor size, overall survival and recurrence in GC patients. **a** Cluster analysis of miRNA expression profiles of GC and the ANTT. **b** Expression level of miR-203 was determined in 100 pairs of GC tissues and their corresponding ANTT by Real-time PCR and normalized to U6. **c** The patients were divided into ANTT, tumor size <5 cm and tumor size >5 cm groups. The diagram showed the miR-203 expression in each group. *P < 0.05. **d**, **e** GC patients were divided into low miR-203 expression group and high miR-203 expression group respectively, according to the result of Real-time PCR. Survival and recurrence curves were drawn with the log-rank test. Results showed the OS and recurrence of GC patients with high or low miR-203 expression

### Low miR-203 expression is related with clinicopathologic features, poor prognosis and recurrence in GC patients

We further examined the association between miR-203 expression and clinicopathological features in GC patients. As shown in Table 1, the results indicated that miR-203 expression was significantly associated with tumor size (*P = 0.006*), but did not correlate with age, sex, vascular invasion and pathological stage in GC patients (*P > 0.05*). Furthermore, we analyzed the relationship between miR-203 expression and GC patients’ prognosis and recurrence. Kaplan-Meier and Multivariate analysis showed that tumor size and miR-203 were the independent factors of the prognosis (Additional file 1: Table S1) and recurrence (Additional file 2: Table S2) in GC patients. Survival curves showed that GC patients with low miR-203 expression had shorter OS (Fig. 1d) and higher recurrence rate (Fig. 1e) than those with high miR-203 expression (Fig. 1d). The 1-, 3-, and 5-year OS rates of GC patients with low miR-203 expression were 81.8 %, 45.5 %, and 14.2 %, respectively, while those with high miR-203 expression were (93.5 %, 66.8 %, and 35.6 %, respectively). The 1-, 3-, and 5-year recurrence rates of the low miR-203 group were 27.9 %, 64.8 %, and 81.3 %, respectively, significantly higher than those of the high miR-203 group (14.5 %, 33.3 %, and 74.2 %, respectively). These results suggested that decreased expression of miR-203 might be associated with poor prognosis and recurrence of GC patients, involved in the progression of GC.

**Table 1:** The correlation of miR-203 expression with clinicopathological characteristics in GC patients

Variable	miR-203		*P* value
	Low	High	
Age (years)			
≤50	33	21	0.644
>50	26	20	
Sex			
Female	22	18	0.509
Male	37	23	
Tumor size (cm)			
≤5	30	32	0.006
>5	29	9	
Vascular invasion			
No	26	21	
Yes	33	20	0.483
Pathological staging			
I/II	25	24	0.114
III/IV	34	17	

### MiR-203 overexpression inhibits proliferation and colony formation and its knockdown promotes cell proliferation in GC cells

Having investigated the correlation of miR-203 expression with tumor size in GC patients (Table 1), we continued to explore the functions of miR-203 in GC growth. In our study, we analyzed the expression levels of miR-203 in a panel of human GC cell lines. The results showed that HGC-27 and BGC-823 cell lines with high malignance displayed lower miR-203 expression levels (Fig. 2a) and were chosen for further functional studies. We used lentivirus-mediated miR-203 overexpression to infect HGC-27 and BGC-823 GC cells (Fig. 2b). Furthermore, we explored the effects of miR-203 overexpression on cellular proliferative functions in GC cells by MTT assay and found that miR-203 overexpression significantly inhibited the growth of HGC-27 and BGC-823 cells (Fig. 2c, d). Colony formation assay shows that miR-203 overexpression decreased cell colony formation in HGC-27 and BGC-823 cells (Fig. 2e, f).

**Fig. 2:** MiR-203 inhibited proliferation and colony formation of GC Cells. **a** Expression levels of miR-203 in a panel of human GC cell lines. **b** The expression level of miR-203 in lentivirus-mediated miR-203 infected GC HGC-27 and BGC-823 cells. **c**, **d** Proliferative activity of GC cells was detected by MTT assay at the indicated time after seeding. **e**, **f** Effect of miR-203 overexpression on colony formation of GC cells. **P < 0.01

Moreover, we found that miR-203 knockdown promoted cell growth (Additional file 3: Figure S1A), but exerted no effect on cell colony formation (Additional file 3: Figure S1B) in MKN-28 and MGC-803 cells with high miR-203 expression. We examined the protein expression levels of PIBF1 and its downstream factors such as Akt, EGFR and STAT3 by Western blotting. The results showed that miR-203 knockdown upregulated the protein expression of PIBF1and p-Akt, but had no effect on the expression of Akt, EGFR and STAT3 in MKN-28 and MGC-803 cells (Additional file 3: Figure S1C).

### PIBF1 is a novel target of miR-203

To uncover the mechanisms by which miR203 affects cell growth in GC, we attempted to identify potential target genes of miR-203. We searched publicly available miRNA-target prediction websites for potential genes under the control of miR-203. Among hundreds of different targets, progesterone immunomodulatory binding factor 1(PIBF1) seemed to be of particular interest. To further confirm whether miR-203 could directly bind to the 3’ UTR of PIBF1, the WT 3’ UTR or the mutant 3’ UTR target sequences (Fig. 3a) were cloned into the luciferase reporter vector, and transfected into cells with a referential vector. Our results showed that miR-203 overexpression suppressed both the mRNA (Fig. 3b) and protein expression level (Fig. 3c) of PIBF1 in HGC-27 and BGC-823 cells. In addition, miR-203 overexpression inhibited the luciferase activity of WT 3’ UTR of PIBF1 in GC cells (Fig. 3d).

**Fig. 3:** MiR-203 inhibited the luciferase activity of WT 3’UTR of PIBF1 and decreased its mRNA and protein expression levels. **a** Diagrams showed the miR-203 putative binding sites and corresponding mutant sites of PIBF1. **b**, **c** The expression level of PIBF1 was tested with Real-time PCR and Western blotting assays in miR-203 and miR-NC groups. **d** Luciferase activity was determined after miR-203 transfection. Data were normalized to the luciferase activity after transfection with miR-NC

### Knockdown of BIBF1 inhibits proliferation and colony formation of GC cells

To further inquire into the cell proliferative functions of BIBF1 in GC cell, MTT and colony formation assays were performed. We found that PIBF1 in HGC-27 and BGC-823 cells was effectively knocked down by PIBF1 shRNA in both the mRNA (Fig. 4a) and protein level (Fig. 4b). Moreover, PIBF1 knockdown significantly reduced the cells proliferation (Fig. 4c, d) and weakened the colony formation capacity in HGC-27 and BGC-823 cells (Fig. 4e, f).

**Fig. 4:** Knockdown of PIBF1 inhibited proliferation and colony formation of GC cells. The expression level of PIBF1 was examined by Real-time PCR (**a**) and Western blotting (**b**) in lentivirus-mediated PIBF1 shRNA infected GC HGC-27 and BGC-823 cells. **c**, **d** Proliferation activity of GC cells was evaluated by MTT assay at the indicated time after seeding. **e**, **f** Effect of PIBF1 knockdown on colony formation of GC cells. **P < 0.01

### MiR-203 suppresses PIBF1-mediated activation of Akt signaling

Studies have shown that PIBF1 plays its role by regulating Akt, EGFR, and STAT3 pathways in cancer cells [3]. To further clarify the molecular mechanism by which PIBF1 contributed to miR-203-induced cell proliferation, lentivirus-mediated PIBF1 was used to transfect into miR-203-treated HGC-27 and BGC-823 cells, indicating that miR-203 depressed cell proliferation via inhibition of the PIBF1 expression (Fig. 5a, c). Furthermore, we examined the protein expression levels of Akt, EGFR and STAT3, which were the potential downstream regulatory factors of PIBF1 related to cell growth by Western blotting. The results showed that miR-203 downregulated the protein expression of p-Akt by inhibition of the PIBF1 expression, but had no effect on the expression of Akt, EGFR and STAT3 (Fig. 5b). Thus, PIBF1 restoration partially counteracted the tumor suppressive effects of miR-203 in GC cells.

**Fig. 5:** PIBF1 overexpression attenuated miR-203-induced inhibition of GC growth and Akt signaling. **a** Lentivirus-mediated PIBF1 overexpression was used to transfect into miR-203-treated GC cells for 72 h, and cell proliferative activity was examined by MTT assay. **b** The protein expression levels of PIBF1 and downstream factors including p-Akt, Akt, EGFR, and STAT3 were detected by western blotting. **c** Lentivirus-mediated PIBF1 was used to transfect into miR-203-treated GC cells for consecutive five days, and cell proliferative activity was examined by MTT assay. **P < 0.01, *P < 0.05

### MiR-203 overexpression inhibited GC growth in vivo

Our findings in vitro indicated that miR-203 overexpression suppressed the growth of GC cells. Therefore, the xenograft tumor model was constructed to validate the tumor growth in vivo. During the whole tumor growth period, the growth activity of GC was measured. The tumors of GC appeared significantly smaller in miR-203 group compared with the miR-NC group (Fig. 6a, b). When the tumors were harvested, the average weight and volumes of the tumors in miR-203 group were significantly smaller than those in si-NC group (**P < 0.01, Fig. 6c, d). IHC staining was used to further evaluate the protein expression of PIBF1, Akt, EGFR and STAT3 in GC tissues. We found that the expression levels of PIBF1 and p-Akt were downregulated in miR-203 group compared with the miR-NC group, and Akt, EGFR and STAT3 had no differential expression between miR-203 and miR-NC group (Fig. 6e).

**Fig. 6:** MiR-203 overexpression inhibited GC growth in vivo. **a** Representative photographs of GC tissues derived from HCG-27-miR-203 or HCG-27-miR-NC cells in nude mice. **b** The growth curve showed that miR-203 inhibited gastric tumor growth compared with the miR-NC group. **c**, **d** At the end of the experiment, the average volume and weight of gastric tumors in miR-203 group were significantly lower than those of the miR-NC group. **e** IHC analysis of the protein expression of PIBF1, p-Akt, Akt, EGFR, and STAT3 in gastric tumors. The data were shown as the means ± SD of three independent experiments. *P < 0.05, image scale: 50 μm

## Discussion

High recurrence rate and rapid tumor growth remain the major cause of increase GC survival rate. Therefore, it is indispensable to gain a better understanding of the mechanisms of GC proliferation. MiRNAs related to tumor proliferation control GC progression and metastasis. Low expression of serum miR-203 is found significantly associated with poor disease-free and overall survival in patients with GC [18] and non-small cell lung cancer (NSCLC) [27]. But, the prognostic significance of miR-203 expression in human GC tissues and its underlying molecular mechanisms have been seldom reported. In the present study, we screened the differentially-expressed miR-203 between GC tissues and the ANTTs and verified that miR-203 expression was significantly downregulated in GC tissues. Then, we found that miR-203 expression was negatively correlated with the tumor size in GC patients and presented the independent risk factors of OS and recurrence rate in GC patients. Our findings suggested that miR-203 might have the potential to serve as a biomarker for prognosis and recurrence in GC patients.

MiRNAs have been fused into carcinogenic programs by regulating genes at post-transcriptional level and involved in tumor development and progression. Evidence shows that miR-203 acts an important role in the regulation of tumor proliferation, migration and invasion. Some studies indicate that miR-203 overexpression suppresses cell growth and metastasis via targeting different genes in different tumor tissues, such as targeting TBK1 in Osteosarcoma [28], ADAM9 and long non-coding RNA HULC in hepatocellular carcinoma [29], Rap1A in prostate cancer [30], Ran and miR-21 in esophageal cancer [31]. However, few studies show that miR-203 may function as the carcinogenic factor via enhancing cell proliferation, migration and invasion by degrading SIK1 in pancreatic cancer [32]. In the present study, we further evaluated the functions and targeted genes of miR-203 in GC cells and found that miR-203 overexpression inhibited cell proliferation and colony formation, while its knockdown promoted cell proliferation in GC cells, indicating miR-203 as a tumor suppressor in GC.

Progesterone-induced blocking factor (PIBF) is an immunomodulatory protein acting the role in the regulation of the immune response in the reproductive system. PIBF1 has been reported overexpressed in various tumors and is correlated with the growth, invasion and metastasis in cancer patients [33, 34]. Our studies showed knockdown of PIBF1 reduced cell proliferation and colony formation, and PIBF1 was predicted to be a direct target of miR-203 by bioinformatics analysis and was validated by western blotting in GC cells. Studies have shown that PIBF1 promotes tumor growth and invasion by regulating Akt, ERK, and STAT3 signaling pathways [35]. We found that miR-203 exerted targeted inhibition of PIBF1 expression and downregulated its downstream p-Akt, its knockdown upregulated the expression of PIBF1 and p-Akt, and the restoration of PIBF1 abrogated the anti-proliferative effects of miR-203 in GC cells, suggesting that miR-203 might inhibit GC proliferation via targeting PIBF1/Akt signaling.

## Conclusions

In conclusion, our findings indicate that decreased expression of miR-203 is associated with tumor size, poor prognosis and recurrence in GC patients, and miR-203 overexpression suppresses the GC growth by targeting PIBF1/Akt signaling, suggesting that miR-203 may have the important therapeutic potential for treatment of GC.

## Additional files

Additional file 1: Table S1. Univariate and Multivariate Analyses of Factors Associated with Overall Survival. (DOC 32 kb) Additional file 2: Table S2. Univariate and Multivariate Analyses of Factors Associated with Cumulative Recurrence. (DOC 32 kb) Additional file 3: Figure S1. MiR-203 knockdown enhanced the proliferation in GC cells. (A) Cell proliferative activity of GC cells was examined by MTT assay at the indicated time after seeding. (B) Effect of miR-203 knockdown on colony formation of GC cells. **P* < 0.05. (C) The protein expression levels of PIBF1 and downstream factors including p-Akt, Akt, EGFR, and STAT3 were examined by western blotting. (TIF 11367 kb)
